# LncRNA CHRF-induced miR-489 loss promotes metastasis of colorectal cancer via TWIST1/EMT signaling pathway

This article has been retracted.

**DOI:** 10.18632/oncotarget.16850

**Published:** 2017-04-05

**Authors:** Youmao Tao, Tao Han, Tao Zhang, Chong Ma, Caixia Sun

**Affiliations:** ^1^ Department of Gastrointestinal Colorectal and Anal Surgery, China-Japan Union Hospital of Jilin University, Changchun 130033, China

**Keywords:** LncRNA CHRF, miR-489, TWIST1/EMT, metastasis, CRC

## Abstract

microRNA-489 (miR-489) is a novel cancer-related miRNAs and functions as a tumor suppressor in human cancers. While, the clinical significance of miR-489 and its role in colorectal cancer (CRC) remain rarely known. Here, we found that the levels of miR-489 in CRC tissues were significantly lower than those in matched tumor-adjacent tissues. Furthermore, decreased levels of miR-489 also observed in CRC cell lines compared to HIEC cells. Clinicopathological analysis revealed that miR-489 underexpression was positively correlated with advanced pT stage, pN stage and AJCC stage. Moreover, miR-489 low expressing CRC patients showed a obvious shorter survival. Functionally, miR-489 restoration inhibited cell migration and invasion as well as epithelial-mesenchymal transition (EMT) in HCT116 cells, while miR-489 loss facilitated these cellular processes in SW480 cells. *In vivo* experiments revealed that miR-489 overexpression reduced the number of metastatic nodules in nude mice liver. Notably, TWIST1 was recognized as a direct downstream target of miR-489 in CRC cells. Interestingly, TWIST1 restoration abrogated the effects of miR-489 on CRC cells with enhanced cell migration, invasion and EMT process. Furthermore, overexpression of long noncoding RNA cardiac hypertrophy-related factor (lncRNA CHRF) was inversely correlated with miR-489 expression in CRC tissues. CHRF knockdown increased the expression of miR-489 and suppressed EMT events of HCT116 cells, while CHRF overexpression showed opposite effects on miR-489 expression and EMT in SW480 cells. Taken together, this work support the first evidence that lncRNA CHRF-induced miR-489 loss facilitates metastasis and EMT process of CRC cells probably via TWIST1/EMT signaling pathway.

## INTRODUCTION

Colorectal cancer (CRC), which ranks fourth in cancer-related deaths, is the third most frequent cancer worldwide [1, 2]. During the last several decades, remarkable advances have been made regarding the early diagnosis and treatment of CRC [3]. However, the long term survival of CRC patients is still poor, especially for those in advanced stages [4]. Most patients in advanced stages were unavailable to effective treatments due to the occurrence of local and systemic metastasis of CRC cells. Unfortunately, the exact mechanisms responsible for the malignant growth and metastatic behaviors of CRC cells remain largely uncovered. Therefore, investigating the molecular mechanisms underlying the growth and metastasis of CRC cells will potentially contribute to identification of novel biomarkers and therapeutic targets of CRC patients.

Epithelial-to-mesenchymal transition (EMT) has been recognized as a main cause for metastasis of CRC by promoting carcinoma invasion and metastasis [5]. The EMT process is very complex and controlled by various families of transcriptional regulators through different signaling pathways, such as Slug, Snail and TWIST1 [5]. TWIST1 plays an essential role in tumor metastasis including CRC [6, 7]. TWIST1 leads to loss of E-cadherin-mediated cell-cell adhesion, increased expression of mesenchymal markers, and induction of cell motility in CRC cells [6, 8]. Recent study reported that miR-381 inhibited migration, invasion and EMT of CRC cells by targeting TWIST1 [9]. Thus, it is worth to investigate novel miRNAs involved in regulation of TWIST1.

MicroRNAs (miRNAs) are a group of small, non-coding, endogenous and single-stranded RNAs that negatively regulate target mRNA for either translational suppression or mRNA degradation [10]. Several studies have reported that miRNAs play pivotal roles in various cellular processes including apoptosis, proliferation, motility and differentiation [11–15]. miR-489 has been found to be underexpressed in breast cancer [16], hypopharyngeal squamous cell carcinoma [17], ovarian cancer [18], lung cancer [19] and hepatocellular carcinoma (HCC) [20]. However, miR-489 is prominently upregulated in oral squamous cell carcinoma [21], clear cell renal cell carcinoma [22, 23], suggesting that the expression and role of miR-489 are variability in different cancers. Our study was aimed to investigated the clinical significance of miR-489 and its underlying mechanisms involved in the progression of CRC.

This study showed that underexpression of miR-489 was correlated with poor prognostic features and reduced survival of CRC patients. We revealed that miR-489 suppressed migration and invasion as well as EMT process of CRC cells. miR-489 that was inversely regulated by long noncoding RNA cardiac hypertrophy-related factor (lncRNA CHRF) exerted an anti-metastatic role probably by targeting TWIST1/EMT signaling pathway. In conclusion, this work supported the first evidence that miR-489 was a potential prognostic biomarker and therapeutic target for CRC.

## RESULTS

### Reduced expression of miR-489 is confirmed in CRC

Eighty CRC tissues and matched tumor-adjacent tissues were detected by qRT-PCR for miR-489 expression. Quantitative data indicated that the levels of miR-489 in CRC tissues were significantly lower than those in matched noncancerous tissues (*P* < 0.05, Figure 1A). In addition, the expressions of miR-489 in five CRC cell lines (HCT116, Caco2, HT29, SW620, SW480) were notably down-regulated compared to a human intestinal epithelial cell line (HIEC) (*P* < 0.05, respectively, Figure 1B). Thus, miR-489 is found to be inhibited during the carcinogenesis of CRC.

**Figure 1:** The expression and prognostic significance of miR-489 in CRC (**A**) miR-489 expression differences between CRC tissues and matched tumor-adjacent tissues. *n* = 80, *P < 0.05 by *t* test. (**B**) Relative expression of miR-489 in five CRC cell lines (HCT116, Caco2, HT29, SW620 and SW480) and a normal human intestinal epithelial cell line (HIEC) detected by qRT-PCR. *n* = three independent experiments with similar results, *P < 0.05 by ANOVA. (**C**) and (**D**) CRC patients were divided into miR-489 high expression group (*n* = 40) and miR-489 low expression group (*n* = 40) based on the median level of miR-489 expression. miR-489 low expressing CRC patients showed a significant decreased overall survival and disease-free survival compared to miR-489 high expressing cases. *P* < 0.05 by Log-rank test.

### Clinical significance of miR-489 in CRC patients

CRC patients were divided into miR-489 high expression group and miR-489 low expression group according to the cutoff value, which was defined as the median level of miR-489. Clinical association analysis indicated that the low expression of miR-489 was positively associated with advanced pT stage and pN stage as well as AJCC stage (*P* < 0.05, respectively, Table 1). Notably, survival analysis indicated miR-489 low expressing CRC patients showed a obvious reduced overall survival and disease-free survival compared to miR-489 high expressing cases (*P* < 0.05, respectively, Figure 1C and 1D). These results suggest that miR-489 may act as a promising prognostic marker for CRC patients.

**Table 1:** The correlation between clinicopathological features and miR-489 expression in colorectal cancer

Features		*n*	miR-489 expression		*P*
			Low (*n* = 40)	High (*n* = 40)	
Age (years)	< 65	31	17	14	0.491
	≥ 65	49	23	26	
Sex	Male	41	25	26	0.154
	Female	39	25	14	
Differentiation	Well+Moderate	56	25	31	0.143
	Poor	24	15	9	
Size (cm)	< 5	35	16	19	0.499
	≥ 5	45	24	21	
pT stage	T1 + T2	17	4	13	0.014*
	T3 + T4	63	36	27	
pN stage	N0	46	16	30	0.002*
	N1 + N2	34	24	10	
pM stage	M0	73	34	39	0.108
	M1	7	6	1	
AJCC stage	I + II	44	13	31	< 0.001*
	III + IV	36	27	9	

AJCC: American Joint Committee on Cancer. *Statistically significant.

### miR-489 regulates migration and invasion of CRC cells

As clinical association analysis showed that miR-489 underexpression was positively correlated with more aggressive phenotype of CRC, we speculated that miR-489 might modulate cancer cell migration and invasion. To verify this hypothesis, HCT116 and SW480, which showed the lowest and highest levels of miR-489, respectively, were used for gain- and loss-of-function experiments. miR-489 restoration were performed in HCT116 cells after precursor miR-489 tranfection (*P* < 0.05, Figure 2A). Wound healing assays revealed that miR-489 restoration prohibited migration of HCT116 cells (*P* < 0.05, Figure 2B). In addition, miR-489 overexpression suppressed the invasive ability of HCT116 cells *in vitro* (*P* < 0.05, Figure 2C). Next, miR-489 knockdown was confirmed by qRT-PCR in SW480 cells (*P* < 0.05, Figure 2D). Further experiments revealed that miR-489 knockdown contributed to migration and invasion of SW480 cells (*P* < 0.05, respectively, Figure 2E and 2F). Notably, *in vivo* experiments revealed that miR-489 overexpression reduced the number of metastatic nodules in nude mice liver (*P* < 0.05, Figure 3). Modulating miR-489 expression had no effect on proliferation of CRC cells, as determined by MTT assays (Supplementary Figure 1). These results disclose that miR-489 inhibits the metastasis of CRC via regulating cell migration and invasion.

**Figure 2:** miR-489 regulates migration and invasion of CRC cells (**A**) HCT116 cells that were transfected with precursor miR-489 and scrambled control, respectively, were subjected to qRT-PCR for miR-489 expression. *n* = three independent experiments with similar results, *P < 0.05 by *t* test. (**B**) Wound healing assays indicated that miR-489 overexpression inhibited migration of HCT116 cells. (**C**) The number of invaded cells was reduced after miR-489 restoration in HCT116 cells. *n* = three independent experiments with similar results, *P < 0.05 by *t* test. (**D**) SW480 cells that were transfected with miR-489 inhibitors and scrambled control, respectively, were detected by qRT-PCR for miR-489 expression. *n* = three independent experiments with similar results, *P < 0.05 by *t* test. (**E**) miR-489 loss facilitated the migratory ability of SW480 cells. (**F**) miR-489 knockdown promoted invasion of SW480 cells *in vitro*. *n* = three independent experiments with similar results, *P < 0.05 by *t* test.

**Figure 3:** miR-489 overexpression inhibits liver metastasis of CRC in nude mice HCT116 cells that were transfected with precursor miR-489 or scrambled control were injected to the spleen subcapsular. HE staining revealed that miR-489 overexpression significantly reduced liver metastases of HCT116 cells. *n* = 5, *P < 0.05 by *t* test. Scale bar: 2 mm.

### miR-489 restrains EMT process of CRC cells

EMT evens are central to tumor progression and malignant transformation in CRC [8]. Accordingly, further studies were performed to confirm whether miR-489 regulated EMT process of CRC cells. Interestingly, miR-489 overexpression in HCT116 cells resulted in up-regulation of epithelial marker (E-cadherin) and down-regulation of mesenchymal marker (Vimentin) as well as the morphology of epithelial-like cells (Figure 4A). While, miR-489 loss in SW480 cells decreased E-cadherin expression and increased Vimentin expression, and then led to the morphology of mesenchymal-like cells (Figure 4B). Thus, miR-489 suppresses EMT progression in CRC cells.

**Figure 4:** miR-489 restrains EMT events in CRC cells (**A**) HCT116 cells were transfected with precursor miR-489 and scrambled control, respectively. Western blotting and IF analysis indicated the miR-489 overexpression up-regulated E-cadherin while down-regulated Vimentin. miR-489 overexpressing HCT116 cells showed the morphology of epithelial-like cells. (**B**) SW480 cells that were transfected with miR-489 inhibitors and scrambled control, respectively. miR-489 loss facilitated EMT process and represented the morphology of mesenchymal-like cells.

### miR-489 directly targets and regulates TWIST1 in CRC cells

Thus, to disclose the potential molecular mechanisms involved in the role of miR-489 in CRC cells, we searched for candidate target genes of miR-489 using publicly available databases, including TargetScan and miRanda. TWIST1 was considered as one of the candidates with which miR-489 could bind directly (Figure 5A). Western blotting data revealed that the expressions of TWIST1 protein in CRC cell lines were prominently increased compared to HIEC cells (*P* < 0.05, respectively, Supplementary Figure 2). Luciferase reporter assays demonstrated that miR-489 overexpression notably reduced the luciferase activity of wt 3′-UTR of TWIST1 (*P* < 0.05, Figure 5B). But miR-489 restoration did not affected the luciferase activity of mt 3′-UTR of TWIST1 (Figure 5B). In addition, miR-489 overexpression reduced the levels of TWIST1 mRNA and protein in HCT116 and HT29 cells (Figure 5C and 5D). Eighty CRC tissues were subjected to qRT-PCR for TWIST1 mRNA expression. Spearman's correlation analysis revealed that the levels of miR-489 were inversely correlated with TWIST1 mRNA expression in CRC tissues (*r* = −0.43, *P* < 0.01, Figure 5E). Next, representative immunostaining showed that miR-489 low-expressing CRC tissue showed strong staining of TWIST1 and Vimentin (Figure 6A and 6E), and weak staining of E-cadherin (Figure 6C). While, weak signal of TWIST1 and Vimentin (Figure 6B and 6F), and strong signal of E-cadherin (Figure 6D) were observed in miR-489 high-expressing tumor. Thus, TWIST1 is a direct target of miR-489 in CRC.

**Figure 5:** miR-489 regulates TWIST1 abundance in CRC cells (**A**) The potential miR-489 binding site in wild type (wt) 3′-UTR sequence of TWIST1. The underlined part is the mutant site designed for mutant (mt) 3′-UTR sequence of TWIST1. (**B**) Overexpression of miR-489 decreased the luciferase activity of wt 3′-UTR of TWIST1, while miR-489 overexpression showed no effect on the luciferase activity of mt 3′-UTR of TWIST1 in HCT116 cells. *n* = three independent experiments with similar results, *P < 0.05 by *t* test. (**C**) and (**D**) HCT116 and HT29 cells that were transfected with correspongding miRNA vectors were confirmed by qRT-PCR and immunoblotting for TWIST1 expression. *n* = three independent experiments with similar results, *P < 0.05 by *t* test. (**E**) An inverse correlation between the levels of miR-489 and TWIST1 mRNA expression was observed in CRC tissues. *n* = 80, *P* < 0.01 by Spearman's rank correlation test.

**Figure 6:** Representative immunohistochemical staining of TWIST1, E-cadherin and Vimentin in CRC tissues CRC tissues were subjected to immunohistochemical staining for TWIST1, E-cadherin and Vimentin expression. miR-489 low-expressing CRC tissue showed strong staining of TWIST1 and Vimentin (**A** and **E**), and weak staining of E-cadherin (**C**). While, weak signal of TWIST1 and Vimentin (**B** and **F**), and strong signal of E-cadherin (**D**) were observed in miR-489 high-expressing tumor. Scale bar: 100 μm.

### TWIST1 restoration abolishes the effects of miR-489 in CRC cells

We next investigate whether miR-489 inhibits migration and invasion as well as EMT process of CRC cells by targeting TWIST1. As expected, re-expression of TWIST1 abrogated the inhibitory effect of miR-489 on EMT process with decreased expression of E-cadherin and increased expression of Vimentin in HCT116 cells (Figure 7A). In addition, the migratory and invasive abilities of HCT116 cells that were reduced by miR-489 overexpression were sequentially rescued by TWIST1 restoration (*P* < 0.05, Figure 7B and 7C). Hence, these results further confirmed that miR-489 inhibits migration, invasion and EMT process of CRC cells probably by targeting TWIST1.

**Figure 7:** TWIST1 restoration abolishes the effects of miR-489 in CRC cells (**A**) miR-489 overexpressing HCT116 cells were transfected with TWIST1 expression vector. TWIST1 overexpression abrogated the inhibitory effects of miR-489 on EMT process. (**B**) TWIST1 re-expression promoted migration of miR-489 overexpressing HCT116 cells. (**C**) TWIST restoration facilitated invasion of miR-489 overexpressing HCT116 cells. *n* = three independent experiments with similar results, *P < 0.05 by ANOVA.

### miR-489 is negatively regulated by lncRNA CHRF in CRC cells

Previous studies have reported that miR-489 is regulated by lncRNA CHRF [24, 25]. Next, our data revealed the levels of CHRF in CRC tissues were notably higher than those in matched tumor-adjacent tissues (*P* < 0.05, Figure 8A). Spearman correlation analysis revealed that the levels of CHRF were inversely correlated with miR-489 expression in CRC tissues (*r* = −0.54, *P* < 0.01, Figure 8B). Furthermore, CHRF expression was knocked down by a specific siRNA in HCT116 cells (*P* < 0.05, Figure 8C). CHRF knockdown increased the expression of miR-489 in HCT116 cells (*P* < 0.05, Figure 8D). Moreover, CHRF overexpression led to a notable reduction of miR-489 in SW480 cells (*P* < 0.05, Figure 8E and 8F). Then, we investigated whether CHRF regulated TWIST1 expression and EMT in CRC cells. Interestingly, CHRF knockdown inhibited TWIST1 expression and EMT progression in HCT116 cells (Figure 9A and 9B). On the contrary, CHRF overexpression promoted TWIST1 expression and EMT process in SW480 cells (Figure 9C and 9D). Thus, lncRNA CHRF contributes to TWIST1/EMT signaling pathway in CRC cells possibly by negatively regulating miR-489.

**Figure 8:** LncRNA CHRF negatively regulates miR-489 expression in CRC (**A**) CHRF expression differences between CRC tissues and matched tumor-adjacent tissues. *n* = 80, *P < 0.05 by *t* test. (**B**) An inverse correlation between the levels of miR-489 and CHRF expression was observed in CRC tissues. *n* = 80, *P* < 0.01 by Spearman's rank correlation test. (**C**) HCT116 that were transfected with CHRF siRNA or scrambled siRNA were detected by qRT-PCR. *n* = three independent experiments with similar results, *P < 0.05 by *t* test. (**D**) CHRF knockdown significantly increased the expression of miR-489 in HCT116 cells. *n* = three independent experiments with similar results, *P < 0.05 by *t* test. (**E**) SW480 cells that were transfected with CHRF vector or empty vector were confirmed by qRT-PCR. *n* = three independent experiments with similar results, *P < 0.05 by *t* test. (**F**) CHRF overexpression notably reduced the expression of miR-489 in SW480 cells. *n* = three independent experiments with similar results, *P < 0.05 by *t* test.

**Figure 9:** LncRNA CHRF induced miR-489 loss promotes EMT process of CRC cells (**A**) CHRF knockdown reduced the expressions of TWIST1 and Vimentin, while increased E-cadherin expression in HCT116 cells. (**B**) CHRF knockdown contributed to the morphology of epithelial-like cells in HCT116 cells. (**C**) CHRF overexpression increased the levels of TWIST1 and Vimentin, while reduced E-cadherin expression in SW480 cells. (**D**) CHRF overexpression facilitated the EMT process of SW480 cells.

## DISCUSSION

The expression status and role of miR-489 in human cancers is a controversial topic. Thus, further study is necessary performed to investigate the clinical significance and role of miR-489 in CRC. In the present study, the expressions of miR-489 in the CRC tissues were prominently lower than those in the matched tumor-adjacent tissues. Furthermore, our data suggest that underexpression of miR-489 was positively associated with advanced pT stage and pN stage as well as AJCC stage. Additionally, we supported the first evidence that underexpresion of miR-489 conferred a obvious poor prognosis of CRC patients. Thus, miR-489 potentially functions as a prognostic marker in CRC.

Underexpression of miR-489 is observed in chemotherapy resistant breast cancer cells [16, 26, 27]. In addition, miR-489 restoration restrains breast cancer cell proliferation, migration and invasion *in vitro* [28]. *In vivo* experiments indicate that miR-489 overexpression prohibits initiation and growth of breast cancer in mice [29]. Furthermore, miR-489 functions as a tumor suppressor in hypopharyngeal squamous cell carcinoma and suppresses growth of cancer cells by targeting protein tyrosine phosphatase, non-receptor type 11 (PTPN11) [17]. Moreover, miR-489 regulates ovarian cancer cell survival, growth and apoptosis via suppression of Akt3 [18]. miR-489 loss promotes invasion and epithelial-mesenchymal transition (EMT) events of lung cancer cells [30]. Recently, the expression miR-489 is found to be down-regulated in HCC tissues, especially in early recurrent cases, and miR-489 underexpression contributes to migration and invasion of HCC cells [20, 31]. Then, we disclosed the biological function of miR-489 in CRC. We demonstrated that miR-489 restoration inhibited migration and invasion as well as EMT of HCT116 cells, while miR-489 loss facilitated theses cellular behaviors of SW490 cells *in vitro*. In addition, reduced the number of metastatic nodules in nude mice liver. These data reveal that miR-489 functions as an anti-metastatic factor by regulating migration and invasion as well as EMT in CRC cells.

EMT events have been widely found in various cancers during metastasis [32]. Many transcriptional factors, including Snail1, ZEB1 and TWIST1 have been implicated in EMT process of CRC cells [33]. Meanwhile, previous studies report that TWIST1 is recognized as a critical regulator of EMT in CRC cells [7, 34]. Notably, we found the miR-489 inversely regulated TWIST1 abundance in CRC cells. Herein, luciferase activity assays indicated that TWIST1 was a direct downstream target of miR-489 in CRC. In addition, an inverse correlation between miR-489 and TWIST1 mRNA expression was observed in CRC tissues. Moreover, TWIST1 restoration abrogated the effects of miR-489 on the migration, invasion and EMT process of CRC cells. Thus, miR-489 inhibits metastasis and EMT of CRC cells probably via targeting TWIST1. Previous studies have reported that miR-489 is regulated by lncRNA CHRF [24, 25]. The expression and role of CHRF in CRC remains unclear. Here, CHRF was overexpressed in CRC tissues compared to matched noncancerous tissues, and was inversely correlated miR-489 expression in CRC tissues. Next, we demonstrated that CHRF inversely regulated miR-489 expression and promotes TWIST1 expression and EMT progression in CRC cells. Taken together, the CHRF-miR-489-TWIST/EMT signaling axis probably exerts key functions in the metastasis of CRC and may represent a therapeutic target for CRC patients.

In conclusion, we show that miR-489 acts as an anti-metastatic factor in CRC. Firstly, our results demonstrate that miR-489 expression was reduced in CRC tissues and cell lines. Then, our clinical data suggest that miR-489 may be used as a novel prognostic marker for CRC patients. Moreover, lncRNA CHRF induced miR-489 loss facilitates migration and invasion as well as EMT probably via targeting TWIST1 in CRC cells. Taken together, our results verify that miR-489 may be served as a potential target for cancer therapeutics in CRC.

## MATERIALS AND METHODS

### Patients

Eighty CRC tissues and matched tumor-adjacent tissues were obtained from the Department of Gastrointestinal Colorectal and Anal Surgery, China-Japan Union Hospital of Jilin University. Tissue specimens were conserved in liquid nitrogen for RNA isolation or 10% formalin for immunostaining until use. No patients received immunotherapy, radiotherapy or chemotherapy before surgery. Tumor staging was based on the American Joint Committee on Cancer (AJCC) staging system (7th edition) [35]. All samples were used after obtaining informed consent. All clinicopathological data of patients were represented in Table 1. The Ethics Committee of Jilin University approved all protocols according to the Declaration of Helsinki.

### Cell culture and transfection

A human intestinal epithelial cell line (HIEC) and CRC cell lines including HCT116, HT29, Caco-2, SW620, and SW480 were bought from American Type Culture Collection (ATCC, Manassas, VA, USA). Cells were cultivated in Dulbecco minimum essential medium (DMEM) (Thermo Fisher Scientific, Waltham, MA, USA) tinting with 10% fetal calf serum (FCS) (Gibco, Grand Island, NY, USA) at 37°C in a humidified atmosphere of 5% CO2.

Precursor miR-489 (HmiR0107-MR04), miR-489 inhibitors (HmiR-AN0528-AM04), and corresponding scrambled control clones (CmiR0001-MR04; CmiR-AN0001-AM04) were purchased, and CHRF siRNA, CHRF expression vector and matched scrambled control vectors were synthesized and purchased from GeneCopoeia^™^ (Guangzhou, China). TWIST1 expression vector and empty vector were obtained from Shanghai Genechem Co., LTD. (Shanghai, China). Vectors were transferred into cells using lipofectamine 2000 (Thermo Fisher Scientific) in accordance with the manufacturer's protocols.

### Quantitative real-time PCR

RNA was isolated using Trizol (Invitrogen, Carlsbad, CA, USA) following the manufacture's protocols. The first strand cDNA was compounded using a Tianscript RT kit (Tiangen biotech, Beijing, China). PCR amplifications for miR-489, CHRF and TWIST1 mRNA were performed with the Kit of TaqMan Human MiRNA Assay (Genecopoeia, Guangzhou, China) and the SYBR Premix Ex Taq^™^ Kit (Takara, Shiga, Japan) in ABI 7300 system (Applied Biosystems, Foster City, CA, USA). U6 and GAPDH were employed as reference genes to normalized the expression of miR-489, CHRF and TWIST1 mRNA, respectively. The primers used for miR-489 and U6 as well as CHRF, TWIST1 and GAPDH were purchased from Sangon Biotech (Shanghai, China).

### Migration and invasion assay

The migratory ability of CRC cells was assessed by wound healing assay. In brief, CRC cells transfected with corresponding vectors were seeded in 6-well plates to form the single confluent cell layer. The wound were made with 100 μL pipette tip in the confluent cell layer. 0 and 48 hours after would scratching, the width of wound was photographed with phase-contrast microscope. We determined the cell invasion capacities by using transwell chambers of pore size 8 μm (coring costar, Cambridge, MA, USA). 24 hours after transfection, 5 × 10^4^ cells were cultured in the 1:9 diluted matrigel-coated (BD Biosciences, Franklin Lakes, NJ, USA) upper chamber with 250 μL serum-free DMEM medium, while 700 μL DMEM medium with 10% fetal bovine serum were added in the lower chamber. After 24 hours, we fixed cells with paraformaldehyde and the cells in upper chamber were removed. Cells in lower chamber were subsequently stained using 0.1% crystal violet solution and photographed.

### Experimental mouse model

Liver metastasis assay in nude mice using the model of subcapsular splenic injection in which the HCT116 cells were injected to the spleen subcapsular. 9 weeks after splenic injection, all mice were sacrificed by cervical dislocation under anesthesia and the livers were obtained. Furthermore, analysis of metastases were assessed on the liver, that was fixed and cut, paraffin-embedded, sectioned and stained for H&E [36]. The protocols for these animal experiments were approved by the Ethics Review Committee of Jilin University.

### Luciferase reporter assay

Wild type (wt) 3′-UTR of TWIST1 was amplified and cloned into pmiR-RB-REPORT^™^ Luciferase. Mutant (mt) 3′-UTR of TWIST1 was constructed by performing mutation on the binding sequences of miR-489. Then, the wt or mt 3′-UTR of TWIST1 and corresponding miRNA vectors were co-transduced into HCT116 cells, respectively. 48 hours after co-transfection, the cells were lysed and detected using a Dual-Luciferase^®^ Reporter Assay Kit (Promega, Madison, WI, USA) based on the manufacturer's protocols.

### Western blotting

Total proteins were collected with RIPA lysis buffer (Santa Cruz Biotechnology, Inc., Santa Cruz, CA, USA) and protein concentrations were measured following the BCA method (Beyotime, Jiangsu, China), and 40ug protein were subjected to 4–20% SDS gel electrophoresis (Sigma) and were then transferred to PVDF membranes (Roche, Indianapolis, IN, USA). Then, 5% milk blocked membranes were incubated with TWIST1 (ab50581, Abcam, Cambridge, MA, USA), E-cadherin (ab1416, Abcam) or Vimentin (ab92547, Abcam) primary antibody and subsequently incubated with matched secondary antibodies (#7074 and #7076, Cell signaling Technology, Beverly, MA, USA). Then, signals for each protein expression were detected with the Bio-Rad Gel imaging system (Bio-Rad, Hercules, CA, USA). GAPDH (G8140, US Biological, Swampscott, MA, USA) was used as a loading control. Alpha Innotech (San Leandro, CA, USA) imaging software was used to quantify western blotting data.

### Immunofluorescence (IF)

CRC cells that transfected with corresponding miRNA vectors were seeded on chamber slides and were fixed with 4% paraformaldehyde for 10 minutes at room temperature. Then, cells were incubated with antibodies against E-cadherin (ab1416, Abcam) or Vimentin (ab92547, Abcam) at 4°C overnight. Then, the slides were incubated with matched secondary antibodies (A16034 and A24517, Invitrogen) at room temperature for 1 hour. The nuclear of EC cells were stained with DAPI (Sigma) at room temperature for 10 minutes. Fluorescence confocal images were captured using a LSM 5 Pascal Laser Scanning Microscope (Zeiss Germany, Oberkochen, Germany).

### Immunohistochemistry (IHC)

The tumor tissues that were previously formalin-fixed and paraffin-embedded were sliced into 4 μm sections, and underwent deparaffination and then rehydration. Antigen retrieval, suppression of endogenous peroxidase activity and 10% skim milk blocking were performed before primary antibody incubation. TWIST1 (ab50581, Abcam), E-cadherin (ab1416, Abcam) and Vimentin (ab92547, Abcam) primary antibodies were used for incubation overnight at 4°C. The slides were then incubated with peroxidase conjugated secondary antibody (ZSGB BIO, Beijing China) for 90 min, and a peroxidase-labeled polymer, DAB solution was used for signal development for 5 min. The sections were counterstained with hematoxylin followed by dehydrating and mounting.

### Statistical analysis

Data were presented as Mean ± SEM and analyzed by GraphPad Prism 5 software (GraphPad Software, Inc, San Diego, CA, USA). Chi-squared test and Spearman's rank correlation coefficient were employed to explore the association between two variables. The Student's *t*-test and ANOVA were carried out to analyze continuous variable. Survival curves were constructed and differences among groups were calculated using the Kaplan-Meier method and Log-rank test. The value of *P* < 0.05 was considered to have statistical significance.

## SUPPLEMENTARY MATERIALS FIGURES AND TABLES


